# Effective Strategies to Promote the Cultivation of Public Legal Consciousness from the Perspective of Social Psychology

This article has been retracted.

**DOI:** 10.1155/2022/8275938

**Published:** 2022-10-03

**Authors:** Liang Yi, Tianxia Li

**Affiliations:** ^1^College of Business, Pingxiang University, Pingxiang, 337055 Jiangxi, China; ^2^Department of Economic Management, Jiangxi Applied Engineering Vocational Institute, Pingxiang, 337042 Jiangxi, China

## Abstract

In order to build a harmonious economic society, show the legal function in the society, enable people to live and work in a better environment, and increase people's practicality in the legal society, it needs to be analyzed from the perspective of social psychology. This paper comprehensively analyzes the current public legal knowledge, uses a deep neural network model, and implements the cultivation of public legal awareness. On this basis, it integrates the data and information before and after 2020, uses the method of book case distribution training, constructs a legal framework, relies on the data distribution technology, constructs a web legal awareness training system, and increases the conditions for promoting the cultivation of public legal awareness based on the background operation of the integrated website. It can be seen that in the perspective of social psychology, the importance of the cultivation of public legal awareness can be achieved through new algorithms, so that people can pay attention to the cultivation of legal awareness, which can provide corresponding protection for the operation and maintenance of the legal system.

## 1. Introduction

The rule of law is an important achievement of human social civilization, and governing the country by law is the socialist development path emphasized by China. The grand goal of governing the country by law requires the public to have a corresponding understanding of socialist law and have a sound legal awareness. Especially for high school students, they should not only put an end to their own illegal acts but also use legal weapons to protect their own rights and interests, and the cultivation of legal awareness has become the key to the construction of the rule of law. This article focuses on the current situation of public legal consciousness and explores the rationalization countermeasures to improve the legal consciousness of high school students, so as to lay the national foundation for the rule of law in China.

Legal consciousness is a kind of social consciousness [1]. It is the individual's subjective state of legal phenomena, the high school students' cognition of the law, their emotions and attitudes towards the law, etc., in view of the differences between the high school students' groups, each high school student's subjective attitude towards the law also varies, which will eventually form differences in legal consciousness. Public legal consciousness is the social public's attitude, psychology, and understanding of the real law. And the evaluation sum of various elements such as beliefs, values, habits, and so on. The function of legal consciousness is mainly reflected in four aspects: first, cognitive function. It mainly aims at understanding the role, nature and characteristics of law. It is the primary embodiment of legal consciousness; second, prediction function [2]. It mainly refers to the individual's experience of predicting the legitimacy of events according to legal norms and whether the prediction behavior is subject to legal sanctions; third, regulation function. Based on the individual's understanding and evaluation of the law, they will adjust their own behavior with the law; fourth, communication function. Legal consciousness will spread through multiple channels and ways and generate corresponding positive energy, which will be carried forward in social groups.  Figure 1 shows the identification diagram of legal awareness cultivation from the perspective of social psychology.

## 2. Current Situation of Public Legal Awareness

### 2.1. Achievements in the Construction of Chinese Public Legal Awareness

With the rapid development of China's social economy, China's politics, law, culture, and other aspects are also making rapid progress. The improvement of material living standards also promotes the public to pay more attention to spiritual literacy [3] and generate relevant legal awareness. Since the 1980s, China has focused on law popularization education, especially for high school students. It is hoped that through education, high school students can contact, understand, and apply the law. Throughout more than 30 years of law popularization education, Chinese citizens in the 21st century have a deeper understanding of basic legal knowledge, legal knowledge, and legal culture [4]. In particular, high school students can adjust their thinking and behavior based on the law and become law-abiding citizens, as shown in Figure 2.

According to relevant data, the crime rate of Chinese high school students has been significantly reduced, which is inseparable from the improvement of legal awareness of high school students [5]. At the same time, most high school students in China can use the law as a weapon to protect their legitimate rights, apply the law to life and study, and protect their own rights and interests with the law. On the premise of the continuous improvement of high school students' legal awareness, the number of criminal cases of high school students shows a downward trend, while the number of rights protection cases is on the rise. Under the domination of legal awareness, high school students use the law to protect their own legitimate rights and interests, which is also the greatest achievement in the construction of Chinese public legal awareness.  Figure 3 shows the protection of their own legitimate rights and interests based on the perspective of social psychology.

### 2.2. Main Problems of Chinese Public Legal Consciousness

Although China has made some achievements in legal awareness [6, 7], there are still many problems. Compared with the development of other fields of consciousness, the development speed of legal consciousness is relatively slow, and there is a certain gap between legal consciousness and the pace of development of the times. Specifically, it is mainly reflected in the following aspects: first, the gap between social public legal consciousness is relatively large. In more than 30 years of law popularization education, high school students have developed legal awareness and know how to use the law as a weapon to protect their own rights and interests, but there are still some high school students with weak legal awareness and do not know how to protect their own rights and interests with the law, and some will also have the phenomenon of fighting and injury, especially in economically backward areas, which is more obvious. Secondly, legal consciousness is framed.  Figure 4 shows the distribution of high school students' legal awareness.

The legal consciousness of Chinese high school students has been negatively influenced by culture for a long time. It hinders the emergence and development of modern legal consciousness and limits the legal consciousness of high school students within the framework. Thirdly, the cultivation of Chinese legal awareness through online channels needs to be improved, as shown in Figure 5 [8].

Although the law popularization education in China has been carried out for more than 30 years, there are still problems of incomplete training, and some legal loopholes are too many and not perfect, which has caused huge obstacles to the cultivation of legal awareness (as shown in Figure 6) [9].

Finally, the legal consciousness of high school students is slowly renewed. Legal consciousness is constantly changing. According to the content of CI system, legal consciousness will be updated with the development of the times and social progress. China's social development is fast, but the renewal of people's legal consciousness is very slow, and there is a large gap between legal consciousness and social development. (as shown in Figure 7) [10].

## 3. Cultivation and Development of Public Legal Consciousness

### 3.1. Gradually Improve the Market Economy System

China should gradually improve the market economic system and promote the legal awareness with economic development. When the mass material base is met, the spiritual needs will be effectively improved. Using a good market economic system to create greater wealth for the society, through the static inspection system helps to enhance the public's legal awareness. (as shown in Figure 8) [11].

On the one hand, to improve the economic level and promote the consciousness of the public in the application of law [12], the government and society should advocate a free economy and allow the public to widely participate in market economic activities. Once the public participates in the market economy, they will face various contradictions and need to solve the contradictions with the help of the law, as shown in Figure 9 [13, 14].

At this time, relevant departments should use legal means to help the public solve contradictions and guide the public to actively study relevant laws, especially high school students, until the public can skillfully use the law as a weapon to protect their own rights and interests (see Table 1 for details) [15].

On the other hand, to cultivate the formation of public legal concepts, the market economic environment requires the public to have the concept of rights, social contract, and law. The government and society should actively cultivate a legal environment. Clear laws and regulations should be used to solve practical contradictions and make the public aware of the importance of law in social life. For example, the government should abandon the traditional mandatory management method and use legal means to manage enterprises. Enterprises also need to carry out corresponding business activities in accordance with the law, and the majority are in enterprises for a long time. With often use of the law to deal with problems, the legal concept will naturally gradually form (the specific questionnaire is shown in Table 2) [16].

### 3.2. Improve the Socialist Democratic System

The social democratic system is closely related to public legal consciousness. A society ruled by law cannot be without democracy, which is the foundation of a society ruled by law. On the one hand, to improve China's democratic system, the democratic system can effectively ensure the public to participate in management activities, ensure the formulation of corresponding laws and regulations in accordance with the interests of the public, and allow the public to participate in the formulation of laws and regulations, thus the public will be more willing to accept the corresponding legal constraints so as to better comply with laws and regulations and carry out activities in accordance with the requirements of laws and regulations. As shown in Figure 10 [17].

In this case, the public's legal awareness will be improved, and they will know how to use the law to protect democratic rights, especially the high school students with high quality [18]. On the other hand, to create a good democratic environment with the development of society, the government has a key influence in social life. The government should create a good democratic environment and supervise the application of rights. Avoid the abuse of judicial power and unfair law enforcement. In a good democratic and legal environment, the public's legal awareness will be further improved, and they will believe more in democracy and the rule of law, as shown in Figure 11 [19].

### 3.3. Enhance the Public's Sense of Legal Security

Law enforcement and strict law enforcement are the key to enhancing the public's sense of legal security. The public's legal awareness is only an understanding of the law in their minds. The transformation of this understanding into reality must rely on strict law enforcement. By only having a high-quality law enforcement team and using the law to protect the legitimate rights and interests of the public, we can enforce the law strictly and fairly, so that the legitimate rights and interests of the public can be effectively protected, so as to enhance the public's sense of trust and security in the law [20, 21]. Once the public has a corresponding sense of security for social law and trusts the protection of their own rights and interests by law, this trust will react on legal awareness and promote the further improvement of public legal awareness, as shown in Figure 12 [22].

### 3.4. Improve the Legal Education Mechanism

Law popularization education is the most direct way to improve public legal awareness, and has been verified in practice. On the one hand, law popularization education is carried out in a diversified way [23]. We should make full use of law popularization education to improve public legal awareness, especially for high school students. To make use of multiple channels and ways to make the public access to legal knowledge, we should not only pay attention to the construction of traditional legal education channels but also use network information channels to carry out legal education, and use websites, WeChat, Weibo, and other tools to carry out legal publicity, so that the public can access legal education anytime and anywhere. On the other hand, close links between law popularization education and life. Law popularization education should pay attention to the update of relevant legal knowledge and content and pay attention to the organic combination with real life. By learning law popularization education, we can solve the practical legal problems and make the public aware of the close connection between law and life, so as to improve their legal awareness, as shown in Figure 13 [24].

## 4. Practical Training Strategies for College Students' Legal Awareness of Innovation and Entrepreneurship

### 4.1. Focus on Building and Improving the Innovation and Entrepreneurship Education Curriculum Education System

In view of the lack of legal awareness-related training courses in the current innovation and entrepreneurship education curriculum system, colleges and universities should correctly understand the relationship between legal awareness and entrepreneurial behavior, think from the perspective of students and comprehensively think about the legal problems that students may face in the practice of innovation and entrepreneurship. On this basis, reasonably determine the content of innovation and entrepreneurship legal education, realize the further improvement of the innovation and entrepreneurship education curriculum system, and truly integrate legal education into innovation and entrepreneurship education, so as to help students master the relevant legal knowledge involved in innovation and entrepreneurship practice and enable students to have the ability to think and solve practical problems by applying legal thinking in innovation and entrepreneurship practice. As shown in Figure 14 [25].

Specifically, colleges and universities need to integrate legal issues and legal cultural knowledge in the fields of innovation and entrepreneurship financing, secured loans, fixed asset leasing, administrative examination and approval, intellectual property rights, and other related fields into innovation and entrepreneurship education, combined with specific examples to help students understand so that students can clarify the relationship between legal knowledge and innovation and entrepreneurship practice. At the same time, colleges and universities should help students understand the contents related to innovation and entrepreneurship activities in the company law, contract law, guarantee law, bill law, and other relevant laws and further enhance students' legal awareness and legal thinking. According to students' professional differences, teachers should pay attention to the application of different cases to help students understand legal knowledge and effectively improve the pertinence and effectiveness of legal awareness training [26].

### 4.2. Cultivate Professional Teachers with Legal Awareness of Innovation and Entrepreneurship

Because the cultivation of legal awareness of innovation and entrepreneurship involves many complex legal knowledge and laws and regulations, teachers who carry out the cultivation of legal awareness must have good legal literacy, otherwise they will be difficult to help students understand the relevant legal knowledge and legal provisions in teaching practice, and they will also be unable to thoroughly understand the content of legal knowledge involved in real cases of innovation and entrepreneurship, as shown in Figure 15 [27].

Therefore, in view of the current lack of professional teachers in the legal awareness training of College Students' innovation and entrepreneurship education, colleges and universities should carry out legal knowledge theme training for teachers. Through training, help them master the legal knowledge related to innovation and entrepreneurship practice, enhance their legal knowledge teaching ability, and ensure that they can truly combine theory with practice in the process of cultivating students' legal awareness so as to effectively help students form a deep understanding and mastery of legal knowledge. At the same time, colleges and universities should pay attention to the introduction of high-quality talents with legal knowledge related professional background and comprehensive practical ability so as to optimize the teaching staff of innovation and entrepreneurship education and effectively improve the level and effectiveness of legal awareness training of innovation and entrepreneurship education, as shown in Figure 16 [28].

### 4.3. Construction of Innovation and Entrepreneurship Legal Services and Legal Aid Base

For college students, even if they have some legal knowledge, they still need to rely on professional legal services and legal aid personnel once they encounter legal problems in the practice of innovation and entrepreneurship due to the lack of legal professionalism. Therefore, colleges and universities need to build innovation and entrepreneurship legal services and legal aid bases, through which students can be provided with free or low-cost legal services and legal aid. In this process, students' legal awareness can be further enhanced, and students can realize the important value and significance of law in resolving risks and solving practical problems. For example, when college students begin to practice innovation and entrepreneurship, due to their lack of corresponding funds, there is often a funding gap when they need legal services, resulting in their inability to obtain effective legal support and assistance. In view of this situation, colleges and universities can strive for the help of social resources, and pay attention to tapping their own resources so as to ensure that college students can obtain sufficient legal services and legal assistance, help them resolve the problems and risks in the practice of innovation and entrepreneurship, and effectively enhance the effectiveness of legal awareness training. At the same time, as China's current judicial assistance system has been relatively perfect, colleges and universities can strive to extend the judicial assistance system to college students' innovation and entrepreneurship practice so as to further ensure that college students can effectively solve the legal problems and risks faced in the process of innovation and entrepreneurship, as shown in Figure 17.

### 4.4. Design and Carry out Practical Application Activities of Innovation and Entrepreneurship Legal Knowledge

Practice is the source of knowledge. In order to effectively cultivate students' legal awareness in the practice of innovation and entrepreneurship education, teachers must pay attention to the design and implementation of practical application activities of innovation and entrepreneurship legal knowledge, so that students can truly understand the practical application fields and specific processes of legal knowledge and master legal knowledge in practice. Therefore, teachers should reasonably carry out the design of practical application activities of legal knowledge from the specific teaching content and the actual characteristics of students, strive to fully mobilize the enthusiasm of students' participation, and promote students to truly form an understanding and mastery of relevant legal knowledge in the process of participating in practical activities. For example, teachers can carry out mock court activities and create situations with the help of real cases related to innovation and entrepreneurship. In this process, students can play different roles in the mock court so as to mobilize students to actively apply relevant legal knowledge. For example, when teaching the contract law, teachers can introduce practical cases about economic contract disputes, let students carry out role-playing and mock court sentencing activities, and enhance students' understanding and mastery of this part of legal knowledge in this process. As shown in Figure 18.

## 5. Based on Legal AI Data and Algorithms, Cultivate Public Legal Awareness

### 5.1. Algorithm Transparency

In the practical application of internal legal AI, the algorithm is usually in a “black box” state for judicial workers. For the accuracy of the algorithm, even in different application scenarios, developers will evaluate their models through F1score, rouge and other indicators, but it seems that they can always find a suitable way to prove the efficiency of their models. The generalization ability of a model needs to be tested by practice. There are many unknowns whether the model developed based on past cases is applicable to current and future cases. For the algorithm itself, developers are often vague about the description of the algorithm, or overestimate it. For the protection of its technical intellectual property rights, developers often do not fully disclose the algorithm, and the fierce market competition has led to legal technology companies often treat their core algorithm or main content confidentially, and the confidentiality of the algorithm may even be supported by the law. In the case of Wisconsin v. Loomis, the defendant believed that there was algorithm discrimination in the algorithm of compass system and requested that the algorithm be made public However, the final decision of the Federal Supreme Court held that the system was neutral and exempted the algorithm developers from the obligation of disclosure. For example, the formula for calculating the compensation amount of medical expenses:

(1) $$\begin{array}{c} A=C+V+B. \end{array}$$

In Formula (1), TCM treatment fee is *A*, the hospitalization fee is *B*, the treatment fee is *C*; and the actual medical cost obtained is *V*. The formula for calculating the compensation amount of work delay is:

(2) $$\begin{array}{c} z=r\left(\frac{\text{yuan}}{\text{day}}\right)\times t\left(\text{day}\right). \end{array}$$

In Formula (2), the compensation amount of delay fee is *z*; the victim's salary is *r*; and the delay time is *t*.

### 5.2. Open Algorithm Source Code

Because there are usually random processes in artificial intelligence algorithms, even if the algorithm is completely transparent, researchers may have many unpredictable changes in the final model results when reproducing the algorithm with different data sets, different parameters, and different training environments. Even if a unified data set, parameter set, and exactly the same training environment are used, the results may be inconsistent due to the internal uncertainty of the algorithm Therefore, some people believe that the requirement of algorithm transparency is superfluous. However, the author believes that the objective difficulties of algorithm recurrence in the above practice should not be the legitimate basis for algorithm nondisclosure. At present, algorithm transparency has become an objective requirement in many scenarios of AI practice. In order to regulate the power of the algorithm and make the developers and users of the algorithm bear relatively balanced risks, the principle of transparency has been paid more and more attention in algorithm development. Because it is difficult to completely eliminate the information asymmetry between developers and users, the principle of transparency can make up for the “digital divide” between decision makers and counterparts, reduce the algorithm monopoly and information monopoly caused by information asymmetry to a certain extent, and then protect the rights of users. For example, the formula for calculating the compensation amount of nursing expenses:

(3) $$\begin{array}{c} G=n\left(\frac{\text{yuan}}{\text{day}}\right)\times t\left(\text{day}\right)*f. \end{array}$$

In formula (3), the compensation for nursing expenses is *G*; the nursing standard is *n*; the nursing period was *t*; the compensation for nursing fee is *f*, and the algorithm flow of the intermediate processing process from input to output is made public so that the decision-making object can fully know and recognize the legitimacy and rationality of the algorithm. Or it can be calculated by:

(4) $$\begin{array}{c} G=\frac{-n\pm \sqrt{t^{2}-4f}}{2n} \end{array}$$

According to the public policy committee of the American computer society, it further refines the transparency of algorithms and puts forward more detailed provisions, such as the principle of knowing, the principle of inquiry and appeal, the principle of algorithm responsibility identification, the principle of interpretation, the principle of data source disclosure, and the principle of auditability. The EU is also actively exploring in this field. According to Article 71 of the General Data Protection Regulation (GDPR), “in any case, appropriate safeguards should be taken, including the right to provide specific information to the data subject and the right to human intervention, so as to express the views of the data subject, obtain the right to interpret the decision and question the decision after evaluation.” It can be seen that how to ensure the transparency and openness of algorithms in practice has become the focus of attention of all countries. The law, which takes the pursuit of fairness and justice as the primary value, will inevitably put forward stricter requirements for the transparency of artificial intelligence algorithms.

### 5.3. Interpretable Legal AI Algorithm

If interpretability is the basic guarantee of the credibility of a legal AI algorithm, then the transparency of the algorithm is the way to realize its credibility. For public authorities such as the court, the transparency of the algorithm is the objective requirement for determining the allocation of responsibility and risk. For researchers, even if there is only a theoretical possibility for the complete reproduction of the model, this does not mean that the need for algorithm transparency is nothing. In addition to the recurrence of the algorithm, the transparency of the algorithm provides a practical basis for others to demonstrate the usability of the algorithm and also facilitates other researchers to conduct more in-depth research on this basis. For the general public, the transparency of the algorithm obviously does not enable them to understand the specific methods adopted by the model and the advantages and disadvantages of the methods, but the legal artificial intelligence technology applied in the public domain, as its users, obviously has the right to know its algorithm. Therefore, the transparency of artificial intelligence judgment algorithm is the key factor for it to obtain the support of the public, courts, and researchers and constantly update and iterate. It shows a series of different graphs of the relationship between the development process of knowledge and structure and uses visualization technology to describe knowledge resources and their carriers, mining, analyzing, constructing, drawing, and displaying knowledge and the relationship between them. Specifically, knowledge atlas is a large-scale, visual semantic network rich in concepts, entities, and relationships, which draws complex domain knowledge through data mining, information extraction, and other technologies. A knowledge map requires a higher degree of granulation of data and models. The finer the model, the more detailed the data, the better the effect of knowledge map. Take dangerous driving cases as an example. Although the cause of action of such cases is simple and the number is huge, the degree of graininess in the knowledge map is still very high, and there are quite a number of factors to be considered, such as death caused by driving after drinking. If this point is ignored, it is difficult to obtain the desired effect by using the knowledge map with low degree of granulation to predict the result of the case.

Knowledge mapping technology can effectively structure legal data, which is also the mainstream direction for many researchers to study the structure of judicial data. However, the development of knowledge atlas involves the intersection of legal knowledge and computer knowledge, and a large number of manual annotations are needed in the early stage of development. At present, when developing the legal knowledge map, relevant institutions often need to recruit a large number of personnel with legal background to manually label, which is also the crux of the current legal knowledge map technology that makes it difficult to achieve leapfrog development. If more scientific and effective research can be carried out in the future and more efficient annotation methods can be adopted, it is reasonable to believe that knowledge atlas technology can enable the structure of legal data so as to promote the leapfrog development of legal artificial intelligence. In the process of developing algorithms, researchers usually give priority to improving the accuracy and rationality of algorithms, or the development idea is “effect oriented”.

The legitimacy of this approach lies in if the artificial intelligence algorithm with a large difference in the matching degree with solving practical problems (such as data set mismatch) is rashly used in judicial practice, the final training result may be an “under fitting” inaccurate model. Such artificial intelligence cannot improve the efficiency of judicial practice, but may interfere with the normal judicial process and affect judicial justice. On the other hand, high accuracy does not mean that the effect must be good but only indicates that the parameters of the training model are more suitable for the characteristics of the test set data. Because the existing artificial intelligence effect evaluation standards mostly rely on the predesigned test set, in a more general scenario, the actual performance of the model may be far from the test results, or even produce errors, that is, it may produce “over fitting” of the model. In the application scenario of legal AI, the “over fitting” of the model means that the mapping law fitted by the model is far more complex than the law familiar to legal experts, which makes it difficult to visualize the correlation between input and output. How to balance the accuracy and rationality of the model in order to get the ideal result is a problem that the developers of artificial intelligence in the field of justice should pay attention to before large-scale application of algorithms.

## 6. Conclusion

In a word, the positive role of developing legal awareness in college students' innovation and entrepreneurship education in promoting students is to form good legal thinking, respect for the law, abide by the law and apply the law, and improve students' comprehensive innovation and entrepreneurship practice ability. Colleges and universities should strengthen their ideological understanding and face up to a series of problems existing in the current innovation and entrepreneurship education, such as the failure to pay due attention to the cultivation of legal awareness, the failure to build a sound innovation and entrepreneurship education curriculum system, and the lack of professional innovation and entrepreneurship legal awareness training in teachers. By implementing a series of strategies, such as building an innovation and entrepreneurship education curriculum education system including legal courses, building innovation and entrepreneurship legal awareness, cultivating professional teachers, carrying out innovation and entrepreneurship legal services, building a legal aid base, and designing and carrying out innovation and entrepreneurship legal knowledge practical application activities, we can effectively promote the solution of the problems and strive to cultivate students to form good legal awareness, legal thinking, and legal literacy so as to promote their innovation and entrepreneurship practice in an orderly manner and promote the full realization of their personal values.

## Figures and Tables

**Figure 1:** Approval chart of legal consciousness cultivation from the perspective of social psychology.

**Figure 2:** 2010-2019 provincial legal literature and art exhibition.

**Figure 3:** Self legal rights and interests protection chart based on the perspective of social psychology.

**Figure 4:** Distribution of high school students' legal awareness.

**Figure 5:** Cultivation of legal awareness of online channels from the perspective of social psychology.

**Figure 6:** Distribution of legal consciousness barriers based on social psychology.

**Figure 7:** CI system content legal awareness creation diagram.

**Figure 8:** Flow chart of static inspection system based on social psychology.

**Figure 9:** Planning diagram for solving legal contradictions based on the perspective of social psychology.

**Figure 10:** Flow chart of activities required by laws and regulations.

**Figure 11:** Legal consciousness assistance from the perspective of social psychology.

**Figure 12:** Punishment chart for illegal acts of grassroots legal service workers.

**Figure 13:** Cultivation of legal consciousness.

**Figure 14:** Change chart of legal thinking ability to think and solve practical problems.

**Figure 15:** Organization chart of legal awareness training activities based on the perspective of social psychology.

**Figure 16:** Legal consciousness cultivation from the perspective of social psychology.

**Figure 17:** Legal issues and risk aversion diagram based on the perspective of social psychology.

**Figure 18:** Legal teaching plan based on the perspective of social psychology.

**Table 1:** List of weight matters of legal consciousness cultivation based on the perspective of social psychology.

Code	Setting basis	Type of power	Applicable object
1	Articles 3, 5, and 33 of the law of the People's Republic of China on the administration of tax collection.	Administrative expropriation	Company
2	Article 9 of the provisional regulations of the People's Republic of China on property tax.	Administrative expropriation	Personal

**Table 2:** Legal consciousness questionnaire based on social psychology.

Number	Survey questions	Reply and proportion
1	Do you think national security has a lot to do with you	A lot/75%
		Not much/25%
2	Whether to attach importance to current affairs and politics	Follow/80%
		Not concerned/20%

## Data Availability

The data that support the findings of this study are available from the corresponding author upon reasonable request.

## References

[1] Ren X., Li C., Ma X. (2021). Design of multi-information fusion based intelligent electrical fire detection system for green buildings. *Sustainability*.

[2] Jayakumar J., Chacko S., Ajay P. (2021). Conceptual implementation of artificial intelligent based -mobility controller in smart city environment. *Wireless Communications and Mobile Computing*.

[3] Liu X., Su Y.-X., Dong S.-L., Deng W.-Y., Zhao B.-T. (2018). Experimental study on selective catalytic reduction of NO by C_3_H_6_ over Fe/Ti-PILC catalysts. *Ranliao Huaxue Xuebao/Journal of Fuel Chemistry and Technology*.

[4] Şahin N. M., Dayan A. (2021). Multicriteria decision-making applications based on generalized Hamming measure for law. *International Journal of Neutrosophic Science*.

[5] Huang R., Yang X. (2022). The application of TiO2 and noble metal nanomaterials in tele materials. *Journal of Ceramic Processing Research*.

[6] Zhang Q. (2021). Relay vibration protection simulation experimental platform based on signal reconstruction of MATLAB software. *Nonlinear Engineering*.

[7] Drace S., Korlat S., Oki R. (2020). When stereotype threat makes me more or less intelligent: the informative role of emotions in effort mobilization and task performance. *British Journal of Social Psychology*.

[8] Chen Y., Tao K., Jiao W., Yang D. (2020). Investigating the underlying social psychology of the innovation adoption in container trucking industry. *Transportation Research Part A Policy and Practice*.

[9] Kim S. C., Hawkins K. H. (2020). The psychology of social media communication in influencing prevention intentions during the 2019 U.S. measles outbreak. *Computers in Human Behavior*.

[10] Barth M., Masson T., Fritsche I., Fielding K., Smith J. R. (2021). Collective responses to global challenges: the social psychology of pro- environmental action. *Journal of Environmental Psychology*.

[11] Sun Q., Polman E., Zhang H. (2021). On prospect theory, making choices for others, and the affective psychology of risk. *Journal of Experimental Social Psychology*.

[12] Huang C. (2020). User's segmentation on continued knowledge management system use in the public sector. *Journal of Organizational and End User Computing (JOEUC)*.

[13] Gorlova E. (2020). Organizational and legal forms of implementation of megascience projects. *Journal of Physics: Conference Series*.

[14] Tnnessen S., Scott A., Nortvedt P. (2020). Safe and competent nursing care: an argument for a minimum standard?. *Nursing Ethics*.

[15] Nisker J., Mykitiuk R., Joseph M. (2020). Obstetricians and gynaecologists lack knowledge of their legal duty to accommodate women with disabilities to receive equal access to health promotion and care. *Journal of obstetrics and gynaecology Canada: JOGC = Journal d'obstetrique et gynecologie du Canada: JOGC*.

[16] Leos-Toro C., Fong G. T., Meyer S. B., Hammond D. (2020). Cannabis health knowledge and risk perceptions among Canadian youth and young adults. *Harm Reduction Journal*.

[17] Frame J. R., Good B., Slinger P., Smith M. P., Marancik D. (2021). Measuring of the effects of a sea turtle conservation education program on children's knowledge and attitudes in Grenada, West Indies. *Ocean & Coastal Management*.

[18] Jacobson H., Carlson A., Lindahl M. (2021). Legal, environmental and economic issues with functional sales - A case of indoor lighting. *Journal of Cleaner Production*.

[19] Li J., Chen D., Yu N., Zhao Z., Lv Z. (2021). Emotion recognition of Chinese paintings at the Thirteenth National Exhibition of Fines Arts in China based on advanced affective computing. *Frontiers in Psychology*.

[20] Hámor-Vidó M., Hámor T., Czirok L. (2021). Underground space, the legal governance of a critical resource in circular economy. *Resources Policy*.

[21] Ayodele B. V., Mustapa S. I., Witoon T., Kanthasamy R., Zwawi M., Owabor C. N. (2021). Radial basis function neural network model prediction of thermo-catalytic carbon dioxide oxidative coupling of methane to c2-hydrocarbon. *Topics in Catalysis*.

[22] Qi A. (2021). Design of a skin cancer diagnosing web application based on convolutional neural network model and chatterbot application programming interface. *Journal of Physics: Conference Series*.

[23] Cheng Y., Morimoto Y. (2021). Triple-stage attention-based multiple parallel connection hybrid neural network model for conditional time series forecasting. *Access*.

[24] Qiu D., Xu H., Luo D., Ye Q., Ding K. (2020). A rainwater control optimization design approach for airports based on a self-organizing feature map neural network model. *PLoS One*.

[25] Irmak E. (2022). Covid-19 disease diagnosis from paper-based ECG trace image data using a novel convolutional neural network model. *Physical and Engineering Sciences in Medicine*.

[26] Ahmad F., Ahmad T. (2021). Content based image retrieval system based on deep convolution neural network model by integrating three-fold geometric augmentation. *Optical Memory and Neural Networks*.

[27] Ren R., Li X. M., Li Z., Li L. H., Huang Y. Y. (2022). Projected change in precipitation forms in the Chinese Tianshan mountains based on the back propagation neural network model. *Journal of Mountain Science*.

[28] Islahuzaman G., Santoso R., Warsito B., Ispriyanti D., Yasin H. (2021). Development of r-shiny interface for implementation of backpropagation neural network model in breast cancer classification. *Journal of Physics: Conference Series*.

